# DETERMINATION OF THE RELATIONSHIP BETWEEN BASAL CELL CARCINOMA AND HUMAN PAPILLOMA VIRUS, BASED ON IMMUNOHISTOCHEMISTRY STAINING METHOD

**DOI:** 10.4103/0019-5154.55629

**Published:** 2009

**Authors:** M Mokhtari, A Mesbah, P Rajabi, M Ail Rajabi, A Chehrei, K Mougouei

**Affiliations:** *From the Department of Pathology and Surgery, Kashani Hospital, Isfahan, Iran.*; 1 *From the Department of Pathology and Surgery Isfahan Medical School, Isfahan, Iran.*; 2 *From the Department of, Alzahra Hospital, Isfahan, Iran.*; 3 *From the Department of, Alzahra Hospital, Isfahan, Iran.*

**Keywords:** *Basal cell carcinoma*, *immunohistochemistry*, *human papilloma virus*

## Abstract

**Background:**

Basal cell carcinoma (BCC) is the most common skin cancer among Caucasians, and in most cases, occurs in the sun-exposed areas. In recent years, in addition to many other etiologies such as exposure to UV radiation, and occasionally xeroderma pigmentosa, burns, tattoos, and pox scars, human papillomavirus (HPV) is also considered to have an etiologic role. Different studies were conducted with varied results in this regard.

**Aims:**

We evaluate this plausible relationship between HPV and BCC by means of immunohistochemistry (IHC) staining method.

**Methods:**

This is an analytic cross-sectional study in which 160 samples were selected randomly consisting of 80 BCC lesions and 80 safe margins. Sampling was done among paraffin-embedded blocks in pathology ward of Kashani and Alzahra hospitals, Isfahan-Iran, from 2004-2007. A section of each block was IHC stained for HPV immunoreactivity (DAKO, Denmark). This was followed by microscopic evaluation in terms of being positive or negative.

**Results:**

Fifty seven point five percent of the samples belonged to men and the others to women. In 10%, HPV marker was positive, both in lesion and margin. In 83.8% neither the lesions nor the margins were immunoreactive for HPV. Only in 5 cases (6.3%) the lesion was positive and the margin was negative for this marker. There was no case of immunoreactivity for HPV marker in margins, while it was negative in lesions. Our study results followed by McNemar analysis did not show a significant relationship between BCC incidence and HPV existence. This was consistent in both genders (*P* > 0.05, power > 90%).

**Conclusion:**

In this study we did not find a significant relationship between BCC and HPV, but based on review of articles it appears that large multicentric studies are to be conducted in this regard.

## Introduction

Basal cell carcinoma (BCC), also known as rodent or mariner's ulcer, is the most common skin cancer among Caucasians and represents approximately 75% of all skin cancers.[1,2] Mortality rates are reported low.[3,4] But occasionally it may grow aggressively which can lead to extensive tissue destruction.[4,5] Metastasis frequency is very low (<0.1%),[2–5] but, at times, has been documented in lymph nodes, lung, bone, and liver.[6–9]

BCCs are commonly subdivided according to their histological appearances. The major histological patterns include: nodular, morpheaform, and superficial types that have different disease outcome.[3]

The risk for BCC development is associated with environmental factors as well as several patient-dependant factors.[1,2] BCCs generally occur on sun-exposed areas of the body[1,2,10,11] and high-risk patients are often fair-skinned with a history of burning, not tanning, when exposed to sunlight.[10,11] Male sex, older age, and more numbers of previous second-degree sunburns are also high-risk factors for BCC development.[1,2,11] Patients with BCC of the trunk are at increased risk of developing multiple BCCs, and these tumors will develop at a faster rate compared with BCCs located elsewhere on the body.[12,13]

Recently, it has been proven that there is an association between smoking and BCC in young women.[14]

Although infection with human papilloma viruses (HPVs) is a major risk factor for several epithelial cancers,[15–19] an etiologic relationship between HPV and keratinocyte cancers, such as squamous cell carcinomas (SCCs) and BCCs, either in immunocompetent[20,21] or in immunosuppressed[20,22] patients, remains unclear.[23–25]

Several authors have suggested an association between infection with the oncogenic types of HPV and development of BCC.[24–27] The involvement of HPV in human skin cancer was demonstrated first in patients with a rare hereditary disease ‘epidermodysplasia verruciformis’ (EV),[28–30] but to date, a causal connection has not been proven between HPV and BCC in the general population. Therefore we decided to evaluate this questionable correlation.

## Materials and Methods

In this analytic cross-sectional study, 160 paraffin-embedded blocks, microscopically diagnosed as BCC by two expert dermatopathologists, and also their safe margins (80 vs. 80 samples, respectively) were analyzed. Safe margin was defined as a part of perilesional skin that had no evidence of involvement by BCC. This group of samples was considered as control group. These samples were selected from patients admitted to pathology wards of Kashani and Alzahra hospitals (Isfahan-Iran), from 2004-2007.

Blocks without sufficient information (age, gender, and lesion location) or without a safe margin following surgery were excluded from our study. Sampling was done randomly in a simple way and then IHC staining was performed briefed as follows.

Four-micron sections were prepared from paraffin blocks and were placed on poly-l-lysin slides. These slides were dried in an oven at 60°C for 60 min followed by deparaffinization and rehydration. At this stage antigen retrieval was performed by heating in Tris/EDTA buffer (pH 8) for 20 min in a microwave oven at 20% of power. Thereafter, the sections were incubated with HPV monoclonal antibody (1:50) for 20 min at room temperature. Neoplastic cells linked to antibody were visualized at the final step using the LSAB method (Link+Strepavidin-HRP from DAKO, Denmark) according to the manufacturers' instructions.

Finally, the stained slides were evaluated microscopically by this study's administrators separately and the results were documented in terms of being immunoreactive (positive) or not for HPV marker. Immunoreactivity is defined as dark-brown staining of neoplastic cell nuclei.We used a paraffin-embedded block of a proven cervical intraepithelial neoplasia (CIN) as a positive control (recommended positive control for HPV marker) and analyzed our results with McNemar chi-square test by the use of SPSS software (version 12).

## Results

Fifty seven point five percent of the studied samples belonged to men and the other 42.5% were of women. The average age was 64.2 (62.15-66.35) years. The most prevalent tumor locations, the mode groups, were face and nose (33.8 and 23.8%, respectively). On the other hand, the least locations were eyelids and auricles (10 and 15% in sequence) [Table 1]. HPV positive cases in nose and face samples were the most prevalent ones (38.5 and 23.1%, respectively), and on the contrary, it was the least in neck samples (7.7%). Eight cases (10%) were immunoreactive, both in the lesion and margins for HPV; but, in 67 cases (83.8%) the results were negative either in the lesions or in the margins. In five cases of the studied samples (6.3%) HPV was positive in the lesions but negative in margins. Forty percent (40%) of those five cases (with immunoreactive lesions but nonimmunoreactive margins for HPV) were nose samples, followed by one case each of face, neck, and eyelid samples. We found no case in which lesion was not immunoreactive for HPV, while the margin immunoreactive [Tables 1 and 2]. Results were also analyzed in women and men separately [Table 3]. Our findings based on McNemar analytic test failed to demonstrate a significant relationship between BCC and HPV. This is also true for both genders (*P* > 0.05, power > 90%).

**Table 1:** The location of basal cell carcinoma

Percentage	Number	Location
33.8	27	Face
15	12	Ear
17.5	14	Neck
10	8	Eyelid
23.8	19	Nose

**Table 2:** HPV positivity in basal cell carcinoma lesions and their margins

		Margins	
		
		Positive	Negative
BCC lesion	Negative (%)	67 (83.7)	0 (0)
	Positive (%)	5 (6.3)	8 (10)

*P* > 0.05, power > 90%

**Table 3:** HPV positivity in basal cell carcinoma lesions and in their margins in women and men separately

			Margins			
		
			Negative	Positive
BCC lesion	Women	Negative	25	0
			73.5	0
		Positive	4	5
			11.8	14.7
	Men	Negative	42	0
			91.3	0
		Positive	1	3
			2.2	6.5

*P* > 0.05, power > 90%

## Discussion

The human papilloma viruses (HPV) are small viruses with double-stranded DNA that have a particular tropism for the epithelium inducing its proliferation,[31] and can be divided into two groups, mucosal and cutaneous.[32] Although the molecular mechanisms of carcinogenesis by HPV have not been completely elucidated,[31,32] it is apparent that HPV infection is the major risk factor in cervical carcinogenesis.[32]

HPV can produce immortality in keratinocytes and most cervical carcinomas express high-risk E6 and E7 HPV proteins that neutralize cellular tumor suppressor function.[33] In the case of high-risk HPV infection and under favorable conditions, the viral genome is integrated into the host genome, a necessary event for the keratinocytes immortality.[31] During this process the circular viral genome breaks at the level of E1 and E2 regions and never at the level of E6 or E7 regions.[31,32] E6 and E7 function as transforming genes. The E6 protein binds to the tumor suppressor protein p53 and promotes degradation, while E7 protein complexes and inactivates the Rb protein; together, they disrupt cell cycle regulation. E6 and E7 can cooperate with cellular oncoproteins like ras and myc which enable the virus to act at the level of growth factors and cellular and nuclear metabolism producing oncogenic cells. E6 and E7 can induce DNA mutations of the host cell, probably by causing alterations of DNA repair mechanisms. This means that certain types of HPVs are able to cause malignant lesions even without the action of other cofactors.[31]

In general, the relationship between HPV and BCC (compared with those conducted about HPV and SCC) is not well studied. However, the role of HPV infection as a major factor in some epithelial cancers is substantiated,[15–19] but its etiologic role in nonmelanoma skin cancers such as BCC and SCC is still unclear.[23–25] Iftner *et al.*, suggest that high-risk genital HPV types recently identified as significant risk factor for cervical cancer may also represent a risk factor for nonmelanoma skin cancer in a nonimmunosupressed population.[26]

Nortingthon *et al.*, in their study suggest that HPV may play a role in the development of some chronic giant BCCs.[24] The findings of Karagas *et al.*, support a role for HPV types from the genus beta in the pathogenesis of SCC, but not BCC.[23]

Following the analysis of this study results, we observed that the difference between the lesion and the surgical margins in terms of being immunoreactive for HPV was not statistically significant. This difference was also analyzed for each gender, and again no significant difference was seen. Therefore, we thought HPV doesn't play a significant role in development of BCC.

## Conclusion

The study results did not find a significant relationship between HPV existence and BCC development. Such a correlation was neither found in women and men after separate assessments in the present study. But, different and occasionally contradictory results in different studies indicate that large multicentric study is needed for a definite conclusion.
